# Comparison of Wiltse’s paraspinal approach and open book laminectomy for thoracolumbar burst fractures with greenstick lamina fractures: a randomized controlled trial

**DOI:** 10.1186/s13018-018-0743-z

**Published:** 2018-03-02

**Authors:** Zhi-da Chen, Jin Wu, Xiao-tao Yao, Tao-yi Cai, Wen-rong Zeng, Bin Lin

**Affiliations:** Department of Orthopaedics, The 175th Hospital of PLA, the Affiliated Southeast Hospital of Xiamen University, Orthopaedic Center of People’s Liberation Army, No. 279 Zhanghua Road, Zhangzhou, 363000 Fujian People’s Republic of China

**Keywords:** Thoracolumbar burst fractures, Greenstick lamina fractures, Wiltse’s paraspinal approach, Open book laminectomy, Randomized controlled study

## Abstract

**Background:**

Posterior short-segment pedicle screw fixation is used to treat thoracolumbar burst fractures. However, no randomized controlled studies have compared the efficacy of the two approaches––the Wiltse’s paraspinal approach and open book laminectomy in the treatment of thoracolumbar burst fractures with greenstick lamina fractures.

**Materials and methods:**

Patients with burst fractures of the thoracolumbar spine without neurological deficit were randomized to receive either the Wiltse’s paraspinal approach (group A, 24 patients) or open book laminectomy (group B, 23 patients). Patients were followed postoperatively for average of 27.4 months. Clinical and radiographic data of the two approaches were collected and compared.

**Results:**

Our results showed the anterior segmental height, kyphotic angle, visual analog scale (VAS) score, and Smiley-Webster Scale (SWS) score significantly improved postoperatively in both groups, indicating that both the Wiltse’s paraspinal approach and open book laminectomy can effectively treat thoracolumbar burst fractures with greenstick lamina fractures. The Wiltse’s paraspinal approach was found to have significantly shorter operating time, less blood loss, and shorter length of hospital stay compared to open book laminectomy. However, there were two (2/24) patients in group A that had neurological deficits postoperatively and required a second exploratory operation. Dural tears and/or cauda equina entrapment were subsequently found in four patients in group B and all two patients of neurological deficits in group A during operation. No screw loosening, plate breakage, or other internal fixation failures were found at final follow-up.

**Conclusions:**

The results demonstrated that either of the two surgical approaches can achieve satisfactory results in treating thoracolumbar burst fractures in patients with greenstick lamina fractures. However, if there is any clinical or radiographic suspicion of a dural tear and/or cauda equina entrapment pre-operation, patients should receive an open book laminectomy to avoid a second exploratory operation. More research is still needed to optimize clinical decision-making regarding surgical approach.

**Electronic supplementary material:**

The online version of this article (10.1186/s13018-018-0743-z) contains supplementary material, which is available to authorized users.

## Background

Burst fractures are a common form of spinal trauma in the thoracolumbar region, accounting for approximately 60% of thoracolumbar fractures and 10–20% of all spinal fractures [1–3]. Burst fractures are usually caused by high-impact accidents, such as motor vehicle accidents or falls, and are associated with pain, deformity, paralysis, and loss of function [4]. With the increase of high-energy injuries in recent years, the morbidity rate from thoracolumbar burst fractures is rising (Additional file 1).

When thoracolumbar burst fractures occur, injury to the anterior and middle aspects of a vertebral segment arises, the severity of which depends on both complex anatomy and the distinct mechanism of injury [5, 6]. Often, there is a loss of height at the anterior aspect of the vertebral body and posterior retropulsion of bony fragments into the spinal canal. This may occur with or without fractures in the lamina. When a lamina fracture occurs, it may be complete or incomplete (greenstick fracture) and may be accompanied by dural tears or cauda equina entrapment [5]. Posterior retropulsion of bony fragments does not always cause a neurological deficit owing to the large dimensions of the spinal canal in the thoracolumbar region. However, previous reports have shown a significant relationship between cauda equina entrapment and neurological deficits [7–10]. Surgical reduction can close a lamina fracture and entrap nerve roots (Additional file 2). However, it is not always possible to determine by pre-operative clinical and radiography examination whether a patient with a thoracolumbar burst fracture and accompanying greenstick lamina fracture has dural tears and/or cauda equina entrapment in the absence of neurological deficits [11, 12].

Management of thoracolumbar burst fractures with accompanying greenstick lamina fractures aims to reduce the fractures, relieve spinal cord compression, reconstruct spine stability, and restore correct alignment. Although various treatment strategies have proven effective for treatment of thoracolumbar burst fractures [13, 14], debate remains regarding optimal treatment when there is an associated greenstick lamina fracture. Despite the lack of a standardized treatment approach, it is generally accepted that posterior short-segment pedicle screw fixation is superior to conservative management due to its excellent three-dimensional stability [15]. The Wiltse’s paraspinal approach through the gap between the multifidus and longissimus muscles has shown satisfactory results for treatment of thoracolumbar fractures [16]. However, performing an open book laminectomy allows for direct visualization of dural tears and cauda equina entrapment and prevents neurological deficit postoperatively. Nevertheless, there is a lack of clinical evidence directly comparing the Wiltse’s paraspinal approach with open book laminectomy for treating patients with thoracolumbar burst fractures with greenstick lamina fractures. The present study aimed to directly compare the therapeutic efficacy of the two approaches both immediately postoperatively as well as through longitudinal follow-up.

## Patients and methods

### Clinical data

This prospective, comparative case series was approved by the Institutional Review Board of Xiamen University. Written informed consent was obtained from all patients preoperatively. Forty-seven consecutive patients (31 males, 16 females) who met the following inclusion and exclusion criteria were enrolled in the study between January 2008 and May 2013. Inclusion criteria included (1) single level thoracolumbar burst fractures with greenstick lamina fractures, (2) load sharing classification (LCS) ≥ 6 and/or Thoracolumbar Injury Classification and Severity Score (TLICS) ≥ 4 need the posterior surgical treatment, (3) age between 18 and 56 years, (4) absence of neurological deficit, (5) good general condition for surgical treatment, and (6) spinal canal compromise ≥ 30%. Exclusion criteria were (1) thoracolumbar burst fractures associated with other fractures, (2) extreme age (younger than 18 years, older than 56 years), (3) neurological deficit, (4) surgical contraindications like heart, liver, and kidney dysfunction. The causes of thoracolumbar burst fractures included traffic accidents in 17 cases (36%), falls in 25 cases (53%), and others in 5 cases (11%). The average age was 37.1 years (range, 21–56 years). Patients were randomized according to their sequence of admission to receive either Wiltse’s paraspinal approach (group A, 24 patients) or open book laminectomy (group B, 23 patients). All patients were diagnosed with thoracolumbar burst fracture by clinical symptomatology, thoracolumbar X-ray, three-dimensional (3D) computer tomography (CT), and magnetic resonance imaging (MRI). Study participants were evaluated postoperatively every 3 months. The average duration of follow-up was 27.4 months (range, 18–32 months). Detailed information of clinical parameters is shown in Table 1.

**Table 1:** Detailed information of the patients

No. of patients	
Male [*n* (%)]	31 (66)
Female [*n* (%)]	16 (34)
Age [year (range)]	37.1 (21–56)
Follow-up [month (range)]	27.4 (18–32)
Etiology	
Traffic accidents [*n* (%)]	17 (36)
Fall from the height [*n* (%)]	25 (53)
Others [*n* (%)]	5 (11)

### Operative approach

Each operation (Wiltse’s paraspinal approach or open book laminectomy) had four surgeons. The main surgeon is Dr. Bin Lin, and the attending assistants are Dr. Zhi-da Chen, Jin Wu, and Xiao-tao Yao.

#### Group A––Wiltse’s paraspinal approach

Wiltse’s paraspinal approach was performed as described in previous studies [16]. After epidural anesthesia, the patient was placed in the prone position. A longitudinal median skin incision was made, and the thoracolumbar fascia was opened 2–3 cm lateral to the spinous process. After passing between the multifidus and latissimus muscles, the inferior and superior articular processes and part of the vertebral lamina were removed using a high-speed drill. Routine pedicle screws (Medtronic, Inc., Minneapolis, MN, USA) were inserted bilaterally at the level of the injury and the adjacent levels above and below. Postural reduction was performed by hyperextending the posterior longitudinal ligament. Next, the screws were tightened and autogeneic iliac bone was inserted into the posterolateral bone groove. To ensure that the screw and bone were appropriately fixed, intraoperative radiographs were taken. Finally, the wounds were rinsed and the incisions were closed.

#### Group B––open book laminectomy

Each patient underwent general endotracheal anesthesia and was placed in the prone position. A longitudinal median skin incision was made, and the paraspinous muscles were dissected to expose the spinous processes and vertebral laminae. After laminectomy, there was direct visualization of the dural sac and nerve roots. If there was a visible dural tear or nerve root entrapment, it was repaired and reduced. Posterior segmental stabilization was achieved using pedicle screws after reduction.

### Postoperative management

All patients received intravenous antibiotics for 24 h postoperatively. The drainage tube was removed on postoperative day 2. Patients in group A were placed on strict bed rest for a minimum of 3 days following surgery, patients in group B were placed on bed rest for 1–2 weeks following surgery. And both of them were then allowed to ambulate wearing a thoraco-lumbar-sacral brace. Use of a brace was continued for an average of 8–10 weeks postoperatively.

### Outcome measures

Clinical assessments were performed immediately after surgery. Patients completed regular follow-up every 3 months in the outpatient clinic. The duration of follow-up ranged from 18 to 32 months, with an average of 27.4 months. Frankel grade was used to evaluate function before and after treatment. Furthermore, radiographs, CT, and MRI of the thoracolumbar spine were obtained for all patients immediately postoperatively and every 3 months thereafter. Achievement of union was determined by formation of continuous bony trabeculae of fusion levels as Suk et al. reported [17]. Clinical parameters included operative time, blood loss, average hospital stay, VAS, SWS, complications, and neurologic status (by Frankel grade). Cauda equina notch sign (CENS) [7], anterior segmental height, kyphotic angle, and bony fusion status were assessed with imaging.

### Statistical analysis

All the data are presented as mean ± standard deviation (SD). Statistical significance was determined by Wilcoxon Rank Sum test or unpaired *t* test using the SPSS17.0 program (SPSS Inc., Chicago, IL, USA) with *P* <  0.05 being statistically significant.

## Results

### Clinical parameters and disease characteristics

Table 2 summarizes the patients’ clinical parameters and disease characteristics. Group A consisted of 14 males and 10 females with a mean age of 36.5 ± 8.9 years; mean length of hospital stay was 4.0 ± 0.8 days. The levels involved included T10 (2 cases), T12 (4 cases), L1 (5 cases), L2 (6 cases), and L3 (7 cases). Group B contained 17 males and 6 females with a mean age of 38.3 ± 9.6 years; mean length of hospital stay was 4.6 ± 1.1 days. The levels involved were T10 (2 cases), T11 (2 cases), T12 (4 cases), L1 (4 cases), L2 (6 cases), and L3 (5 cases). There were no differences in sex, age, length of hospital stay, and levels involved between the two groups.

**Table 2:** Clinical parameters and disease characteristics of patients

Group	Sex (M/F)	Age (years)	Involved level						Treatment	Operation time (mins)	Blood Loss (ml)	VAS		Average stay (days)	Complication (%)
			T10	T11	T12	L1	L2	L3				Pre-op	post-op		
A	14/10	36.5 ± 8.9	2	0	4	5	6	7	WPA	65.6 ± 7.7	79.6 ± 27.8	6.2 ± 1.2	2.5 ± 1.2	4.0 ± 0.8	25.0 (3/24)
B	17/6	38.3 ± 9.6	2	2	4	4	6	5	OBLA	126.8 ± 12.7	508.2 ± 125.6	6.3 ± 1.2	3.2 ± 0.9	4.6 ± 1.1	8.7 (2/23)
*P* value	0.260	0.506	0.788						–	< 0.0001	< 0.0001	0.785	0.026	0.065	0.672

*WPA* Wiltse’s paraspinal approach, *OBLA* open book laminectomy approach. *P* < 0.05, significant difference

The mean duration of surgery in group A was 65.6 ± 7.7 min compared to the mean duration for group B of 126.8 ± 12.7 min. This difference was statistically significant (*P* <  0.0001). The mean blood volume loss during surgery was also significantly different between the two groups, with a mean loss of 79.6 ± 27.8 ml in group A and 508.2 ± 125.6 ml in group B. Significant improvement of postoperative VAS scores compared with preoperative scores was observed in both groups. Additionally, statistical analysis found there was a significant difference in postoperative VAS scores between group A and group B (*P* <  0.0001).

### Radiologic assessments

The anterior segmental height was measured on lateral radiography pre- and postoperatively. The mean preoperative anterior segmental height significantly increased postoperatively and remained stable at a 6-month follow-up in both groups (both *P* values < 0.05). However, there was no difference in postoperative anterior segmental height between the groups. Preoperative to immediate postoperative mean angle of kyphotic curvature increased in group A from 21.7 ± 3.9°(range, 11–32°) to 8.4 ± 2.5°(range, 3–18°) and in group B from 20.9 ± 4.2°(range, 12–33°) to 7.2 ± 2.9°(range, 2–14°) (all *P* <  0.05). At a 6-month follow-up, mean kyphotic curvature in both groups was stable compared to immediate postoperative measures. There was no statistical difference in postoperative kyphotic angle between the two groups. Patients in group A had successful bony fusion at a mean of 3.8 ± 0.9 months after surgery compared to 4.6 ± 0.8 months after surgery in group B; this difference in time to bony fusion was significant (*P* < 0.05). Detailed data was showed in Table 3. And in our series of 47 patients, CENS was found in 9 (19%) patients on their MRI examination.

**Table 3:** Radiologic assessments of patients at preoperation, postoperation, and a 6-month follow-up

Group	Vertebral height loss (%)			Kyphotic angle (°)			Bony fusion (months)
	Preoperation	Postoperation	Follow-up	Preoperation	Postoperation	Follow-up	
A	33.8 ± 7.3	8.2 ± 3.4	8.7 ± 3.7	21.7 ± 3.9	8.4 ± 2.5	9.3 ± 2.7	3.8 ± 0.9
B	34.2 ± 6.1	6.5 ± 3.8	6.7 ± 3.5	20.9 ± 4.2	7.2 ± 2.9	9.1 ± 4.2	4.6 ± 0.8
*P* value	0.846	0.133	0.063	0.507	0.154	0.813	0.004

*P* < 0.05, significant difference

### Complications

Of the 24 patients in group A, 2 (8.3%) showed postoperative signs of cauda equina syndrome and neurogenic bladder. One patient with Frankel grade D, another is Frankel grade C. All 2 of these patients received immediate reoperation with open book laminectomy and had improvement in neurological function at a 3-month follow-up. Among them, one patient with first postoperative Frankel grade D had complete recovery of neurological function, while one patient with first postoperative Frankel grade C only recovered to Frankel grade D at a 6-month follow-up.

Surgical complications occurred in 3 patients. One patient in group A had pedicle screws that penetrated approximately 3 mm beyond the anterior edge of the vertebral body. Two patients in group B acquired a superficial infection, which healed following debridement. However, no screw loosening, plate breakage, or other internal fixation failures were found at final follow-up.

### Functional outcome

Functional outcomes were assessed using SWS scores. In group A, 19 cases were classified as excellent and 5 cases were classified as good. In group B, 20 cases were labeled excellent and 3 cases were marked as good. No statistical differences were observed in SWS functional outcomes between the two groups.

Typical cases are shown in Fig. 1 (case 3), Fig. 2 (case 21), and Fig. 3 (case 37).

**Fig. 1:** Preoperative, postoperative, and follow-up radiographs of the patient who had thoracolumbar burst fractures with greenstick lamina fractures managed by the open book laminectomy approach (case 3). **a**–**e** X-ray, CT, and MRI before the posterior pedicle screw fixation. **f**–**h** X-ray and CT at 3 days after operation. **i**, **j** MRI at 3 months after operation. **k**, **l** CT at 6 months follow-up

**Fig. 2:** Preoperative, postoperative, and a 3-month follow-up radiographs of a patient with thoracolumbar burst fractures and greenstick lamina fractures treated with the open book laminectomy approach (case 21). **a**–**d** X-ray, CT, and MRI before operation. **e**–**g** X-ray and CT at 3 days after operation. **h**, **i** X-ray at a 3-month follow-up

**Fig. 3:** Preoperative, postoperative, and intra-operative graphs of a patient with thoracolumbar burst fractures and greenstick lamina fractures treated with the Wiltse’s paraspinal approach (case 37). **a**–**e** X-ray, CT, and MRI before the pedicle screw fixation. **f**–**j** X-ray, CT, and MRI after operation. The patient appeared neurological deterioration postoperatively and was offered immediately open book laminectomy surgical treatment. **k**–**o** X-ray, CT, and MRI after re-operation. **p** Dural tears and cauda equina entrapment existed in the patient

## Discussion

### Clinical features of greenstick lamina fractures in thoracolumbar fracture

Due to its special biomechanical characteristics, thoracolumbar spine is the most common region where spine trauma occurs. Usually, the presence of laminar fractures indicates a more severe injury of thoracolumbar spine [18]. Although the clinical characteristics and treatment strategies for thoracolumbar spine fractures have been largely reported [13, 14], few studies have reported on thoracolumbar fractures combined with a greenstick lamina fracture. Consequently, the features and treatment strategies of this particular type of fracture are far from clear. The presence of laminar fractures in the thoracolumbar burst fractures indicates a high rate of dural sac and neural element trapping. The association between dural tears and burst fractures was first reported by Miller et al. [10]. They documented the existence of dural tears and cauda equina entrapment in patients with thoracolumbar burst fractures associated with the separation of pedicles and pointed out that neural elements were often entrapped between the fracture fragments of lamina. Then, this type of incomplete laminar fracture was described as greenstick fracture of the anterior cortex of the lamina that occurred secondary to splaying of the posterior arch of the vertebra under axial loading [19]. Currently, the injuries have been well demonstrated with CT scan and MRI. Burst fractures can cause the pedicles and posterior elements of the vertebral column to fracture laterally, which may lead to retropulsion of the bone from the vertebral body and protrusion of the dura between laminar fracture fragments [20]. After dissipation of axial loading, the nerve roots and dura are entrapped. The incidence of greenstick lamina fractures in thoracolumbar fractures is range from 23.3–78.3% [7, 20, 21]. The rate of dural rupture is 19 to 25% [7, 20, 21], and the occurrence of nerve root entrapment is estimated to be approximately 26.1% [7]. In our present study, dural tears and/or cauda equina entrapment were subsequently found in 17.4% (4/23) patients in group B.

Previous study found that cauda equina entrapment occurs in 36–44% of patients with a dural tear, and there is a significant association between a dural tear and neurological deficit [10]. However, no neurological deficit preoperatively does not exclude either a dural tear or cauda equina entrapment because the content and size of the vertebral canal distinguish the thoracolumbar area from other regions [19]. Most of patients with dural tear and nerve root entrapment were neurologically intact before surgery [20]. Therefore, it is crucial to determine whether there is a greenstick lamina fracture before surgery that may be accompanied by cauda equina entrapment. Unfortunately, no radiological guidelines exist for findings on any imaging modality that give adequate sensitivity and specificity for dural tears or cauda equina entrapment in the absence of clinical neurological symptoms on admission [10, 22]. If special attention is not paid to the presence of a greenstick lamina fracture and the possibility of asymptomatic nerve root entrapment, it may lead to serious consequences for these patients. A patient with lumbar burst fracture without neurological deficit before operation developed neurogenic bladder after posterior instrumentation. And then the patient required reoperation during which a dural tear and nerve root were entrapped in the lamina [20]. Although conventional myelography may diagnose a dural tear, myelography may be harmful in a patient with a fracture due to the positioning required to perform the procedure [23]. MR-myelography (MRM) with heavy T2-weighting can achieve similar results to conventional myelography [24]. However, MRM is not routinely available at all hospitals. Lee et al. reported an association between dural tears and certain MRI findings of lamina fractures: an interpedicular distance > 28 mm, a central canal ratio < 0.46, and an acute angle of the retropulsed segment < 135° [25]. However, the number of participants in the analysis was small and the exact measurement of the central canal diameter ratio is difficult. Recently, Yoshiiwa et al. discovered a v-shaped image on transverse T2-weighted MRI where entrapped cauda equina gathers between lamina fractures that they named the CENS [7]. The CENS had only 26% sensitivity for thoracolumbar burst fractures, but 100% specificity for the existence of cauda equina entrapment. However, only 23 patients participated in the study. In our series of 47 patients, only 9 (19%) patients were found to have the CENS on their MRI examination.

### Therapeutic strategies of greenstick lamina fractures in thoracolumbar fracture

Various strategies have been described for the treatment of thoracolumbar burst fractures, including nonoperative and surgical treatment. It was demonstrated in a prospective, randomized study that nonoperative treatment for thoracic and lumbar spine fractures resulted in loss of height of the anterior vertebral column and moderate to severe back pain at long-term follow-up [26]. Alternatively, surgical treatment improves biomechanical stability that allows for correction of kyphosis and fracture reduction [27, 28]. A systematic review of surgical management of thoracolumbar burst fractures suggested that the posterior approach had lower complication rates when compared to anterior or combined approaches [15]. Short-segment posterior pedicle screw fixation including the fractured vertebra has been widely used in recent years. Not only can short-segment posterior pedicle screw fixation including the fractured vertebra partially correct kyphosis and provide earlier pain relief owing to its three-column fixation and quick fusion, but also it can also avoid the need for anterior reconstruction [15, 29, 30]. Both the Wiltse’s paraspinal approach and open book laminectomy achieved satisfactory results for treatment of thoracolumbar burst fractures. Shorter operative time and less blood loss were observed using the Wiltse’s paraspinal approach compared with open book. However, open book laminectomy allows for direct visualization of the dural sac and nerve roots when treating patients in whom dural tears and/or cauda equina entrapment may be a concern. Aydinli et al. proposed that if there is any suspicion of a dural tear and/or nerve root entrapment, a posterior approach with an open book technique should be used to expose the dura safely before any reduction maneuvers are undergone [20]. Similar conclusion was found by Ozturk et al. [31]. To the best of our knowledge, the present study is the first randomized controlled study to compare the Wiltse’s paraspinal approach with open book laminectomy for treatment of thoracolumbar burst fractures with greenstick lamina fractures. In our study, on the basis of the LCS and TLICS, all 47 patients with LCS ≥ 6 and/or TLICS ≥ 4 received posterior short-segment pedicle screw fixation including the fractured vertebra. In addition, good or excellent results were obtained in all 47 patients using SWS functional assessment. And there were 2 patients, all in group A, without preoperative neurological deficit who had neurological deterioration postoperatively. All 2 patients received immediate surgical treatment with open laminectomy. Dural tears and/or cauda equina entrapment were subsequently found in all 2 patients.

Based on our current experience and review of the literature, we know that dural tears and/or cauda equina entrapment are frequently associated with greenstick lamina fractures accompanying thoracolumbar burst fractures. However, it is not always possible to preoperatively determine by clinical and radiography examination whether these complications are present. The Wiltse’s paraspinal approach, while less invasive, does not provide visualization of the dural sac to inspect for tears or cauda equina entrapment. Any operative reduction that closes the lamina fractures may crush the entrapped nerve roots and show symptoms postoperatively (Fig. 4).

**Fig. 4:** The mechanism of thoracolumbar burst fractures with greenstick lamina fractures cause neurological deficits postoperatively. **a**–**b** Dural tears and/or cauda equina entrapment are associated with greenstick lamina fractures accompanying thoracolumbar burst fractures. There is no neurological deficit because the dural sac is loose before reduction. **c**, **d** Any operative reduction that closes the lamina fractures may crush the entrapped nerve roots and show symptoms postoperatively

## Conclusion

To the best of our knowledge, the present study is the first prospective, randomized study to compare the two surgical approaches (Wiltse’s paraspinal approach and open book laminectomy) to treat thoracolumbar burst fractures with greenstick lamina fractures in patients without preoperative neurological deficits. There were no differences in the postoperative anterior segmental height, kyphotic angle, or SWS functional outcome. Open book laminectomy was associated with increased operative time, increased blood loss, prolonged hospital stay, longer time to bony fusion, and increased postoperative VAS scores compared with patients who underwent the Wiltse’s paraspinal approach. When a CENS between the greenstick lamina fracture is detected preoperatively on MRI, or when there is any suspicion for a dural tear and/or cauda equina entrapment, patients are at increased risk of sub-clinical nerve root entrapment and should receive an open book laminectomy to avoid the need for a second exploratory operation.

## Additional files

Additional file 1: Thoracolumbar burst fractures with greenstick lamina fractures. (MP4 1251 kb)

Additional file 2: Closed reduction of greenstick lamina fractures. (MP4 1736 kb)

## Abbreviations

3D: Three-dimensional
CENS: Cauda equina notch sign
CT: Computer tomography
LCS: Load sharing classification
MRI: Magnetic resonance imaging
MRM: Magnetic resonance myelography
SD: Standard deviation
SWS: Salvati and Wilson assessment score
TLICS: Thoracolumbar Injury Classification Score
VAS: Visual analog scale
